The article "Combination of aloin and metformin enhances the antitumor effect by inhibiting the growth and invasion and inducing apoptosis and autophagy in hepatocellular carcinoma through PI3K/AKT/mTOR pathway" was retracted in 2024. Reasons: errors in the data; plagiarized data; plagiarized images; overlap with other authors' work.

# Combination of aloin and metformin enhances the antitumor effect by inhibiting the growth and invasion and inducing apoptosis and autophagy in hepatocellular carcinoma through PI3K/AKT/mTOR pathway

**DOI:** 10.1002/cam4.2723

**Published:** 2019-12-12

**Authors:** Ruijie Sun, Ruiren Zhai, Changlin Ma, Wei Miao

**Affiliations:** ^1^ Department of Hepatobiliary Surgery Jining First People 's Hospital Jining Shandong China; ^2^ Department of Cancer Center Tumor Center Shandong Sunshine Hospital Weifang Shandong China; ^3^ Department of Health Care Jining First People's Hospital Jining Shandong China

**Keywords:** aloin, autophagy, hepatocellular carcinoma therapy, metformin

## Abstract

Hepatocellular carcinoma (HCC) is a devastating and highly metastatic cancer worldwide. Metformin (MET) is the priority drug for treatment of type 2 diabetes; however, it possesses multiple biological effects like anticancer and hepatoprotective activity. Herein, we examined the effects of aloin (barbaloin) and MET as well as combination treatment in HCC cell line in vitro and in vivo. As a result, aloin and MET alone exhibited inhibitory effects on proliferation and invasion of HepG2 and Bel‐7402 cells. Specially, combination treatment of aloin and MET showed enhanced inhibitory effects in vitro. Aloin and MET alone induced apoptosis and autophagy in vitro. Similarly, aloin and MET cooperated to promote apoptosis and autophagy in HepG2 and Bel‐7402 cells. In the HepG2 xenograft models, aloin in combination with MET confine tumor growth and facilitate apoptosis and autophagy. Both the in vitro and in vivo results showed that aloin and MET alone as well as combination treatment activated the PI3K/AKT/mTOR pathway. Overall, our research demonstrated that the concomitant treatment with aloin and MET enhances the antitumor effect by inhibiting the growth and invasion as well as inducing apoptosis and autophagy in HCC through PI3K/AKT/mTOR pathway.

## 1 INTRODUCTION

Hepatocellular carcinoma (HCC) is the most devastating and aggressive form in liver tumor. The HCC incidence continues to increase rapidly, ranking third with more than 600 000 deaths per year.^1^ HCC shows a strong tendency to invade hepatic vessels.^2^ More effort should be made in exploring new therapy strategies for HCC.

Metformin (MET) is the first‐line antidiabetogenic drug for treatment of type 2 diabetes.^3^ More than that, MET was broadly reported for its anticancer effect in recent years.^4^ Besides, MET is able to protect the liver against chemical or viral hepatotoxicants.^5^ Interestingly, MET was reported to combine with aspirin to inhibit HCC growth and metastatic potential in vitro.^6^

Aloin (also named barbaloin) was proved to possess anticancer role in different kinds of cancer cells: Ehrlich ascites carcinoma cell, myeloid leukemia, and acute lymphocytes leukemia cancerous cells.^7^ In addition, aloin was found to suppress gastric cancer and non‐small cell lung cancer,^8^, ^9^ which further confirm the anticancer activity of aloin. Importantly, aloin was able to enhance the anticancer activity of cisplatin B16‐F10 melanoma cells.^10^ In this study, we aim to investigate the enhanced effect of aloin and MET combination treatment on growth, invasion, apoptosis, and autophagy in vitro and in vivo.

## 2 METHODS AND MATERIALS

### 2.1 Cell culture and reagents

The HepG2 cells (American Type Culture Collection) and Bel‐7402 cells were cultured in ATCC‐formulated Eagle's Minimum Essential Medium (EMEM; Gibco). To make the complete growth medium, 10% fetal bovine serum (FBS, Gibco), penicillin (100 units/mL, Gibco), and streptomycin (100 g/mL, Gibco) were supplemented. The cell lines were placed in an incubator with 5% CO_2_ at 37°C. Aloin was obtained from Selleck and dissolved in DMSO (concentration: 1 mg/ml). MET HCl was obtained from Selleck and dissolved in ddH_2_O (concentration: 1 mg/ml).

### 2.2 Cells and animals grouping

HepG2 cells were treated with PBS (phosphate buffer saline) (control), aloin (50 μmol/L^9^), MET (400 μmol/L^11^), and aloin (50 μmol/L)+ MET (400 μmol/L). The cells in all groups were harvested after 48 hour of treatment to measure the expression of corresponding cellular markers.

Bel‐7402 cells were treated with PBS (control), aloin (50 μmol/L), MET (400 μmol/L), and aloin (50 μmol/L)+ MET (400 μmol/L). The cells in all groups were harvested after 48 hours of treatment to measure the expression of corresponding cellular markers.

The orthotopic xenograft mouse models were established on BALB/c athymic nude mice (female, 6‐week‐old), whereas HepG2 xenografts were established by inoculating 2.0 × 10^6^ HepG2 cells into the right flank near the hind leg of each nude mouse. The experiments began when the mice bore palpable tumors (the tumor volume was ~100 mm^3^), and they were randomly divided into four groups (n = 7) with treatment of (a) control (normal saline, every day), (b) aloin (40 mg/kg^9^), (c) MET (200 mg/kg^12^) or (d) aloin (40 mg/kg)+ MET(200 mg/kg). The standard dose of MET for treating humans is 1000 to 2500 mg, usually given twice daily. MET (p.o) was administered at 300 mg/kg in drinking water. This can be translated to the human equivalent dose using the Reagan‐Shaw method.^13^ By the end of the experiment and after the rats were anesthetized, the trunk blood samples were collected from each rat.

### 2.3 Cell growth assay

Cell proliferation was determined by Cell Counting Kit‐8 (CCK‐8) assay. HepG2 and Bel‐7402 cells were pretreated with PBS, 50 μmol/L aloin, 400 μmol/L MET, and aloin (50 μmol/L) + MET (400 μmol/L) for 0, 24, 48, 72, and 96 hours, then cells were detached and seeded into 96‐well plates at a density of 1.5 × 10^3^ cells in 200‐μl complete growth medium/well. Then, the 96‐well plates were cultivated in incubator at 37°C with 5% CO_2_. CCK‐8 experiment was performed according to the manufacturer's instructions. Absorbance at 490 nm was obtained by a microplate reader (BioTek Instruments, Inc).

### 2.4 Colony formation assay

HepG2 and Bel‐7402 cells were pretreated with PBS, 50 μmol/L aloin, 400 μmol/L MET, and aloin (50 μmol/L) + MET (400 μmol/L); cells were cultured in drug‐free medium for approximate 14 days. The cells were fixed with cold methanol‐glacial acetic acid and stained with crystal violet.

### 2.5 Cell invasion assay

Transwell experiment was performed to detect cell invasion of HepG2 cells. HepG2 cells were seeded (5 × 10^4^/200 µL) into the upper transwell chambers with serum‐free DMEM. The lower chambers were filled with 500‐µL 10% FBS EMEM. Simultaneously, PBS (control), 50 μmol/L aloin, 400 μmol/L MET, and aloin (50 μmol/L) + MET (400 μmol/L) were added into upper chamber. After 24‐hours incubation, cells in lower chambers were fixed in 95% ethanol, and then stained with hematoxylin. The invasive number of cells was calculated and imaged under an inverted microscope.

### 2.6 Wound scratch assay

The monolayer cells were scraped in a 6‐well plate using a sterile pipette for a gap of about 1 mm to ensure that there was no cell presence in this gap. HepG2 and Bel‐7402 cells were pretreated with PBS, 50 μmol/L aloin, 400 μmol/L MET, and aloin (50 μmol/L) + MET (400 μmol/L) for 24 hours; cell images in the scratch area were captured under the inverted microscope at 100 × magnification (Tokyo, Japan).

### 2.7 Cell apoptosis assay

Flow cytometry was performed to detect cell apoptosis. As previously described,^14^ HepG2 cells were gently homogenized and harvested. Cells were resuspended in EMEM at a density of 1 × 10^5^, stained with Annexin V‐FITC and PI, respectively. Finally, flow cytometric analysis was performed according to the manufacturers' instructions (Cell Sorter BD FACSAria II, BD Biosciences).

### 2.8 Cell autophagy assay

Cell autophagy was detected by analyzing the protein expression of Beclin‐1, ATG8, P62, and LC3 as well as the location of LC3. Protein expressions were determined by western blotting. The location of LC3 was detected by immunofluorescence staining. The experiment was performed as described by H. Tong et al.^15^ Fluorescence was detected under the confocal microscopy (Nikon C1SiR, inverted microscope Nikon TE200, Image Systems).

### 2.9 Western blotting analysis

Forty microgram proteins extracted from cells and tumors were resolved on (6%‐12%) SDS‐PAGE, then the proteins on gel were transferred to PVDF membranes (Millipore). Next, PVDF membranes were probed with primary antibodies. Antibodies were as follows: anti‐PI3K, AKT and mTOR (Abcam), anti‐GAPDH (Abcam), anti‐Ki67 (Abcam), anti‐Caspase‐3 (Abcam), anti‐VEGF (Abcam), and anti‐MMP‐9 (Abcam). After removing the primary antibody, membranes were incubated with horseradish peroxidase (HRP)‐conjugated secondary antibody (Santa Cruz Biotechnology). The target proteins were visualized using the Amersham ECL Prime Western Blotting Detection Reagent (Amersham Pharmacia Biotech). Finally, protein images were obtained by a ChemiDocxRS imaging system and analyzed by Quantity One analysis software (Bio‐Rad Laboratories).

### 2.10 The xenograft tumor model assay

The orthotopic xenograft models were established according to the study by M.A. Hossain et al.^16^ Mice were divided into four groups: normal saline (control), aloin (40 mg/kg), MET (200 mg/kg), and aloin (40 mg/kg) + MET (200 mg/kg). Each group had six mice. In aloin (40 mg/kg) and aloin (40 mg/kg) + MET (200 mg/kg) groups, mice were injected with aloin (40 mg/kg) intraperitoneally 1 day after the injection of tumor cells three times a week. In MET (200 mg) and aloin + MET groups, mice were injected with MET (200 mg/kg) intraperitoneally 1 day after the injection of tumor cells three times a week. All animals were sacrificed at the 30th day; median survival of the nice and tumor weight were measured.

### 2.11 Immunohistochemistry assay

The paraffin‐embedded tumor sections were incubated with anti‐Ki67 and anti‐VEGF (Abcam). The immunohistochemistry assay was performed as previously described by N. D et al.^17^

### 2.12 Statistics analysis

SPSS software (version 19.0) was used for all the statistical analyses. The data were shown as mean ± SD. Statistical comparisons were analyzed by one‐way analysis of variance (ANOVA) followed by the least significant difference (LSD) test. The difference was considered statistically significant when values of *P* < .05.

## 3 RESULTS

### 3.1 Aloin, MET, and combination inhibited cell proliferation in vitro

As shown in Figure 1, the effects of MET and aloin  on HepG2 and Bel‐7402 cell proliferation were confirmed by CCK‐8 assay (Figure 1A,B) and colony formation assay (Figure 1C). Both aloin and MET alone inhibited the proliferation of HepG2 and Bel‐7402 cells compared with the control (*P < *.05). In addition, the combination treatment of aloin and MET showed that the proliferation‐inhibiting effects were stronger in HepG2 and Bel‐7402 cells compared with the MET alone group (*P < *.05). The proliferation result was verified by protein expression of Ki67 and PCNA exhibited in Figure 1. The relative expression of Ki67 and PCNA was markedly suppressed in HepG2 and Bel‐7402 cells by aloin and MET alone (*P < *.05). Similarly, combination of aloin and MET showed that the expression of Ki67 and PCNA was less than MET alone (*P < *.05).

**Figure 1:** Aloin, MET, and combination inhibited cell proliferation in vitro. A, HepG2 cells were treated with PBS, MET (400 μmol/L), aloin (50 μmol/L), and combination treatment (MET 400 μmol/L and aloin 50 μmol/L), the CCK‐8 assay was used to determine cell viability. B, Bel‐7402 cells were treated with PBS, MET (400 μmol/L), aloin (50 μmol/L), and combination treatment (MET 400 μmol/L and aloin 50 μmol/L), the CCK‐8 assay was used to determine cell viability. C, Effects on the colony formation in HepG2 and Bel‐7402 cells were determined for 24 h. D, Relative protein expression of Ki67 and PCNA was detected by western blotting in HepG2 cells. The representative column diagrams showing results of relative protein expression. E, Relative protein expression of Ki67 and PCNA was detected by western blotting in Bel‐7402 cells. The representative column diagrams showing results of relative protein expression. Date are represented as the mean ± SD of three independent experiments. *P < .05,**P < .01, compared with Control,*^#^P* < .05, compared with MET

### 3.2 Aloin, MET, and combination inhibited invasion in vitro

As shown in Figure 2, the effects of MET and curcumin on HepG2 and Bel‐7402 invasive cells were confirmed by transwell chambers assay (Figure 2A,B) and wound‐healing assay (Figure 2C,D) . Both aloin and MET alone decreased the invasive HepG2 cell number compared with the control (*P < *.05). Expectedly, the combination treatment of aloin and MET reduced the invasive cells in HepG2 and Bel‐7402 compared with the MET alone (*P* < .05). The relative expressions of MMP‐9 and VEGF were significantly reduced in HepG2 and Bel‐7402 cells by both aloin and MET alone treatment (*P* < .05). Also, the expressions of MMP‐9 and VEGF were reduced in combination therapy than MET alone (*P* < .05).

**Figure 2:** Aloin, MET, and combination inhibited cell invasion in vitro. A, Cell invasion of HepG2 was analyzed by Transwell assay (magnification, ×400). B, Cell invasion of Bel‐7402 was analyzed by Transwell assay (magnification, ×400). C, Effects on the wound healing in HepG2 cells were determined for 0 and 24 h (magnification, ×100). D, Effects on the wound healing in Bel‐7402 cells were determined for 0 and 24 h (magnification, ×100). E, The protein expression of MMP‐9 and VEGF was detected by western blotting in HepG2 cells. The representative column diagrams showing results of relative protein expression. F, The protein expression of MMP‐9 and VEGF was detected by western blotting in Bel‐7402 cells. The representative column diagrams showing results of relative protein expression. Date are represented as the mean ± SD of three independent experiments. *P < .05, **P < .01, compared with Control,*^#^P* < .05, compared with MET

### 3.3 Aloin, MET, and combination promoted apoptosis in vitro

As shown in Figure 3A, the apoptotic HepG2 and Bel‐7402 cells were increased both aloin and MET alone compared with the control (*P* < .05); meanwhile, the combination of aloin and MET significantly increased the apoptotic cell compared with the MET alone (*P* < .05). The expression of cleaved caspase‐3 and caspase‐9 was significantly increased in HepG2 and Bel‐7402 cells by both aloin and MET alone treatment (*P* < .05); interestingly, the expression of cleaved caspase‐3 and caspase‐9 was high in combination therapy than MET alone (Figure 3B, *P* < .05).

**Figure 3:** Aloin, MET, and combination promoted cell apoptosis in vitro. A, Apoptosis of HepG2 cells was detected by flow cytometry. The representative column diagrams showing results of number of Q2 + Q4 as apoptotic cells. B, The protein expression of cleaved caspase‐3 and caspase‐9 was detected by western blotting in HepG2 cells. GAPDH was used as control. The representative column diagrams showing results of relative protein expression. C, Apoptosis of Bel‐7402 cells was detected by flow cytometry. The representative column diagrams showing results of number of Q2 + Q4 as apoptotic cells. D, The protein expression of cleaved caspase‐3 and caspase‐9 was detected by western blotting in Bel‐7402 cells. GAPDH was used as control. The representative column diagrams showing results of relative protein expression. Date are represented as the mean ± SD of three independent experiments. *P < .05, **P < .01, compared with Control,*^#^P* < .05, compared with MET

### 3.4 Aloin, MET, and combination induced autophagy in vitro

As shown in Figure 4, both aloin and MET alone increased the relative expressions of autophagy‐promoting proteins including Beclin‐1, LC3II, and ATG8 in HepG2 and Bel‐7402 cells compared with control, with reduced relative expression of P62 (*P* < .05). Interestingly, combination therapy showed the expression level of P62 was less but the expression of Beclin‐1, LC3II, and ATG8 was high in HepG2 and Bel‐7402 cells than MET alone (*P* < .05). As shown in Figure 4, both aloin and MET alone increased the LC3‐positive puncta per cell in HepG2 and Bel‐7402 cells. Similarly, combination therapy exhibited more LC3‐positive puncta per cell than MET alone (*P* < .05).

**Figure 4:** Aloin, MET, and combination promoted cell autophagy in vitro. A, The protein expression of autophagy‐related markers was detected by western blotting in SepG2 cells. GAPDH was used as the control. The representative column diagrams showing results of relative protein expression. B, The protein expression of autophagy‐related markers was detected by western blotting in Bel‐7402 cells. GAPDH was used as the control. The representative column diagrams showing results of relative protein expression. C, LC3 (green) in HepG2 cells was detected by immunocytochemistry. DAPI (blue) = nuclei. The representative column diagrams showing the LC3‐positive puncta per cell. D, LC3 (green) in Bel‐7402 cells was detected by immunocytochemistry. DAPI (blue) = nuclei. The representative column diagrams showing the LC3‐positive puncta per cell. Date are represented as the mean ± SD of three independent experiments. *P < .05, **P < .01, compared with Control,*^#^P* < .05, compared with MET

### 3.5 Aloin, MET, and combination inhibited the PI3K/AKT/mTOR pathway

As shown in Figure 5, both aloin and MET alone as well as combination treatment reduced the phosphorylation levels of PI3K, AKT, and mTOR significantly in HepG2 and Bel‐7402 cells compared with control (*P* < .05); meanwhile, combination treatment of aloin and MET showed stronger inhibition of the phosphorylation levels of PI3K, AKT, and mTOR compared with MET alone (*P* < .05).

**Figure 5:** Aloin, MET, and combination inhibited the activation of PI3K/AKT/mTOR pathway in vitro. A, The protein expression of PI3K/AKT/mTOR and p‐PI3K/p‐AKT/p‐mTOR was detected by western blotting in SepG2 cells. GAPDH was used as the control. The representative column diagrams showing results of relative protein expression. B, The protein expression of PI3K/AKT/mTOR and p‐PI3K/p‐AKT/p‐mTOR was detected by western blotting in Bel‐7402 cells. GAPDH was used as the control. The representative column diagrams showing results of relative protein expression. Date are represented as the mean ± SD of three independent experiments. *P < .05, **P < .01, compared with Control, *^#^P* < .05, compared with MET

### 3.6 Aloin, MET, and combination suppressed the tumor growth in vivo

As shown in Figure 6A, both aloin and MET alone as well as combination treatment significantly decreased the xenograft tumor weight. Consequently, both aloin and MET alone as well as combination treatment increased the survival of nude mice (Figure 6B). In addition, both aloin and MET alone as well as combination treatment inhibited the expression of Ki67 and VEGF obviously (Figure 6C). Consistent with the in vivo results, both aloin and MET alone as well as combination reduced the expression of Beclin‐1 and LC3II as well as the phosphorylation levels of PI3K, AKT, and mTOR markedly (Figure 7A‐B).

**Figure 6:** Aloin, MET, and combination suppressed the tumor growth in vivo. A, Nude mice bearing subcutaneous xenograft HepG2 were treated with PBS, 200 mg/kg MET alone, 40 mg/kg Aloin alone, and combination treatment (200 mg/kg MET + 40 mg/kg Aloin). A, The tumor weight was determined when the mice were killed at the 30th day. B, The survival of mice was determined every 2 d for 30 d. C, Immunohistochemistry analysis of expression of Ki67 and VEGF (magnification, ×400). D, The representative column diagrams showing results of positive cells (brown). Date are represented as the mean ± SD of three independent experiments. *P < .05, **P < .01, compared with Control, ^#^ *P* < .05, compared with MET. The results were analyzed by one‐way ANOVA followed by the least significant difference (LSD) test

**Figure 7:** Aloin, MET, and combination suppressed the tumor autophagy and PI3K/AKT/mTOR pathway in vivo. A, The protein expression of autophagy‐related markers was detected by western blotting. GAPDH was used as the control. The representative column diagrams showing results of relative protein expression. B, The protein expression of PI3K/AKT/mTOR and p‐PI3K/p‐AKT/p‐mTOR was detected by western blotting. GAPDH was used as the control. The representative column diagrams showing results of relative protein expression. Date are represented as the mean ± SD of three independent experiments. *P < .05, **P < .01, compared with Control, ^#^ *P* < .05, compared with MET

## 4 DISCUSSION

HCC is an aggressive tumor characterized by highly proliferative and invasive capability.^18^ It is meaningful to find more effective medication for HCC therapy. Single‐agent treatment of cancer may produce chemoresistance, dramatically, a large number of studies have shown that combination therapy may have a stronger killing effect on cancer cells. For instance, aloin was reported to enhance the antineoplastic activity of cisplatin B16‐F10 melanoma cells.^10^ Besides, MET and curcumin combination treatment inhibited the growth, metastasis, and angiogenesis of HCC.^19^ Rosiglitazone and MET combined to inhibit HCC.^20^ In present study, we demonstrated that MET in combination with aloin suppress HCC in vitro and in vivo.

Aloin, a natural bioactive anthracycline, is extracted from Aloe barbadensis Miller leaves.^21^ A large number of articles have shown the anti‐inflammatory, antimicrobic, antioxidant, and anticancer potentials.^9^ Till now, we first demonstrated the anti‐HCC effect of aloin. MET was proved to suppress HCC alone or in combination with other medication.^6^, ^19^, ^22^, ^23^In the present study, both aloin and MET alone exhibited anticancer role in HCC. Specially, we demonstrated that aloin and MET alone inhibited the HCC in vitro and in vivo. Logically, aloin and MET alone promoted the apoptosis and autophagy of HepG2 and Bel‐7402 cells in vitro. Besides, aloin in combination with MET showed that proliferation/invasion‐inhibiting and apoptosis/autophagy‐promoting roles were enhanced in HepG2 and Bel‐7402 cells. The result indicates that MET alone has stronger anticancer effect than aloin alone; however, aloin combined with MET exhibits better anticancer effect than MET alone. The results may suggest that aloin enhances the chemosensitivity of MET in HCC. MET is a promising candidate to fight with various cancer including triple‐negative breast cancer;^4^ our experiments suggested that aloin might have additive effect with MET in vitro and in vivo.

PI3K/Akt pathway is associated with cell proliferation, apoptosis, autophagy, and inflammation.^24^ mTOR, an important downstream regulator in the PI3K/Akt pathway, plays an essential role in protein synthesis and autophagy.^25^ Growing evidences have identified that many factors inhibit HCC via inactivation of the PI3K/Akt/mTOR signaling pathway.^26^, ^27^, ^28^ In our in vitro and in vivo results, the PI3K/Akt/mTOR signaling pathway was inhibited, especially in the combination treatment group. The result evidenced that the concomitant treatment with aloin and MET reduced the phosphorylation level of PI3K, AKT, and mTOR.

Autophagy, an intracellular lysosomal pathway, is involved in protein degradation and organelle degradation. Autophagy is closely connected to a variety of human disease and physiology, including HCC.^29^ According to previous study, combination treatment of MET and sorafenib could suppress proliferation and induce autophagy of HCC cells through targeting the mTOR.^12^ In this research, MET was proved to promote autophagy in HepG2 and Bel‐7402 cells and in tumors. Meanwhile, the concomitant treatment with aloin and MET enhanced the cell autophagy.

Autophagy is a mechanism by which the cells try to survive while apoptosis is a mechanism of cell death. Autophagy and apoptosis are two distinct processes which play seemingly opposite biological roles in response to genotoxic or pharmacological stresses. However, both autophagy and apoptosis may be triggered by common upstream signals, resulting in the activation of combined autophagy and apoptosis. Specially, the p38 and JNK MAPK pathways in regulating the balance of autophagy and apoptosis will hopefully provide prospective strategies for cancer therapy.^30^ Interestingly, there is a conflicting report regarding the potential role of p38 MAPK and autophagy. p38 MAPK was found to play a vital role in the switch from autophagy to apoptosis in MS‐275‐induced human colon cancer cells. High expression of p38 induced cell autophagy, but low expression resulted in apoptosis.^31^ Importantly, treatment with MET and sorafenib alleviates endometrial hyperplasia in polycystic ovary syndrome by promoting apoptosis via synergically regulating autophagy.^32^ Furthermore, proapoptotic roles of autophagy have been reported.^33^ Therefore, autophagy and apoptosis might be mutually regulated after treatment to achieve anticancer effects.

In summary, aloin was demonstrated to enhance the anticancer effect of MET via attenuating the proliferation and invasion, and facilitating apoptosis and autophagy in vitro and in vivo. Therefore, aloin is promising to be a novel medication for HCC therapy when combined with MET.

## AUTHOR CONTRIBUTIONS

Ruijie Sun conceived and designed the experiments; Ruijie Sun and RuirenZhai performed the experiments; Changlin Ma analyzed the data; Wei Miao drafted or revised the manuscript.

## References

[1] Siegel RL , Miller KD , Jemal A . Cancer statistics. CA Cancer J Clin. 2018;2018(68):7‐30.10.3322/caac.2144229313949

[2] Jiang JF , Lao YC , Yuan BH , et al. Treatment of hepatocellular carcinoma with portal vein tumor thrombus: advances and challenges. Oncotarget. 2017;8:33911‐33921.2843061010.18632/oncotarget.15411PMC5464922

[3] Ben Sahra I , Le Marchand‐Brustel Y , Tanti J‐F , Bost F . Metformin in cancer therapy: a new perspective for an old antidiabetic drug? Mol Cancer Ther. 2010;9:1092‐1099.2044230910.1158/1535-7163.MCT-09-1186

[4] Lee J , Yesilkanal AE , Wynne JP , et al. Effective breast cancer combination therapy targeting BACH1 and mitochondrial metabolism. Nature. 2019;568:254‐258.3084266110.1038/s41586-019-1005-xPMC6698916

[5] Iranshahy M , Rezaee R , Karimi G . Hepatoprotective activity of metformin: a new mission for an old drug? Eur J Pharmacol. 2019;850:1‐7.3075386910.1016/j.ejphar.2019.02.004

[6] Da A , As S , Wf E‐H , Dm A . Targeting AMPK, mTOR and β‐catenin by combined metformin and aspirin therapy in HCC: an appraisal in Egyptian HCC patients. Mol Diagn Ther. 2018;22:115‐127.2909428710.1007/s40291-017-0307-7

[7] El‐Shemy HA , Aboul‐Soud MA , Nassr‐Allah AA , Aboul‐Enein KM , Kabash A , Yagi A . Antitumor properties and modulation of antioxidant enzymes' activity by Aloe vera leaf active principles isolated via supercritical carbon dioxide extraction. Curr Med Chem. 2010;17:129‐138.1994147410.2174/092986710790112620

[8] Wang Y‐R , Yang S‐Y , Chen G‐X , Wei P . Barbaloin loaded polydopamine‐polylactide‐TPGS (PLA‐TPGS) nanoparticles against gastric cancer as a targeted drug delivery system: studies in vitro and in vivo. Biochem Biophys Res Comm. 2018;499:8‐16.2953496210.1016/j.bbrc.2018.03.069

[9] Zhang Z , Rui W , Wang Z‐C , Liu D‐X , Du L . Anti‐proliferation and anti‐metastasis effect of barbaloin in non‐small cell lung cancer via inactivating p38MAPK/Cdc25B/Hsp27 pathway. Oncol Rep. 2017;38:1172‐1180.2865629310.3892/or.2017.5760

[10] Tabolacci C , Rossi S , Lentini A , et al. Aloin enhances cisplatin antineoplastic activity in B16–F10 melanoma cells by transglutaminase‐induced differentiation. Amino Acids. 2013;44:293‐300.2213940910.1007/s00726-011-1166-x

[11] Vacante F , Senesi P , Montesano A , Paini S , Luzi L , Terruzzi I . Metformin counteracts HCC progression and metastasis enhancing KLF6/p21 expression and downregulating the IGF. Axis. 2019;2019:1‐14.10.1155/2019/7570146PMC635058530774659

[12] Ling S , Song L , Fan N , et al. Combination of metformin and sorafenib suppresses proliferation and induces autophagy of hepatocellular carcinoma via targeting the mTOR pathway. Int J Oncol. 2017;50:297‐309.2795938310.3892/ijo.2016.3799

[13] Shankaraiah RC , Callegari E , Guerriero P , et al. Metformin prevents liver tumourigenesis by attenuating fibrosis in a transgenic mouse model of hepatocellular carcinoma. Oncogene. 2019;38:7035‐7045.3140989610.1038/s41388-019-0942-z

[14] Ferretti AC , Hidalgo F , Tonucci FM , et al. Metformin and glucose starvation decrease the migratory ability of hepatocellular carcinoma cells: targeting AMPK activation to control migration. Sci Rep. 2019;9:2815.3080902110.1038/s41598-019-39556-wPMC6391381

[15] Tong H , Zhu Y , Liu Y . Incidence and risk of fatigue in cancer patients treated with MET inhibitors: A systematic review and meta‐analysis. Medicine (Baltimore). 2019;98:e15522.3114527310.1097/MD.0000000000015522PMC6709275

[16] Hossain MA , Kim DH , Jang JY , et al. Aspirin induces apoptosis in vitro and inhibits tumor growth of human hepatocellular carcinoma cells in a nude mouse xenograft model. Int J Oncol. 2012;40:1298‐1304.2217906010.3892/ijo.2011.1304PMC3584583

[17] Nahari D , Satchi‐Fainaro R , Chen M , et al. Tumor cytotoxicity and endothelial Rac inhibition induced by TNP‐470 in anaplastic thyroid cancer. Mol Cancer Ther. 2007;6:1329‐1337.1743111110.1158/1535-7163.MCT-06-0554

[18] Huang J , Zheng C , Shao J , Chen L , Liu X , Shao J . Overexpression of eEF1A1 regulates G1‐phase progression to promote HCC proliferation through the STAT1‐cyclin D1 pathway. Biochem Biophys Res Comm. 2017;494:542‐549.2907918710.1016/j.bbrc.2017.10.116

[19] Zhang H‐H , Zhang Y , Cheng Y‐N , et al. Metformin incombination with curcumin inhibits the growth, metastasis, and angiogenesis of hepatocellular carcinoma in vitro and in vivo. Mol Carcinog. 2018;57:44‐56.2883360310.1002/mc.22718

[20] Wang X , Chen X , Zhou H , et al. The long noncoding RNA, LINC01555, promotes invasion and metastasis of colorectal cancer by activating the neuropeptide, neuromedin U. Med Sci Monit. 2019;25:4014‐4024.3114467510.12659/MSM.916508PMC6559001

[21] Js Z , Yy H , Th Z , et al. Natural phosphodiesterase‐4 inhibitors from the leaf skin of Aloe barbadensis Miller. Fitoterapia. 2015;100:68‐74.2544942610.1016/j.fitote.2014.11.018

[22] Bhat M , Yanagiya A , Graber T , et al. Metformin requires 4E‐BPs to induce apoptosis and repress translation of Mcl‐1 in hepatocellular carcinoma cells. Oncotarget. 2017;8:50542‐50556.2888158210.18632/oncotarget.10671PMC5584165

[23] Casadei Gardini A , Faloppi L , De Matteis S , et al. Metformin and insulin impact on clinical outcome in patients with advanced hepatocellular carcinoma receiving sorafenib: validation study and biological rationale. Eur J Cancer. 2017;86:106‐114.2898557910.1016/j.ejca.2017.09.003

[24] Nakagawa A , Sullivan KD , Xue D . Caspase‐activated phosphoinositide binding by CNT‐1 promotes apoptosis by inhibiting the AKT pathway. Nat Struct Mol Biol. 2014;21:1082‐1090.2538366610.1038/nsmb.2915PMC4256149

[25] Chen H , Qu Y , Tang B , Xiong T , Mu D . Role of mammalian target of rapamycin in hypoxic or ischemic brain injury: potential neuroprotection and limitations. Rev Neurosci. 2012;23:279‐287.2275278510.1515/revneuro-2012-0001

[26] Li TT , Zhu D , Mou T , et al. IL‐37 induces autophagy in hepatocellular carcinoma cells by inhibiting the PI3K/AKT/mTOR pathway. Mol Immunol. 2017;87:132‐140.2843389010.1016/j.molimm.2017.04.010

[27] Wang SS , Chen YH , Chen N , et al. Hydrogen sulfide promotes autophagy of hepatocellular carcinoma cells through the PI3K/Akt/mTOR signaling pathway. Cell Death Dis. 2017;8:e2688.2833314210.1038/cddis.2017.18PMC5386547

[28] Kim J , Jiang J , Badawi M , Schmittgen TD . miR‐221 regulates CD44 in hepatocellular carcinoma through the PI3K‐AKT‐mTOR pathway. Biochem Biophys Res Commun. 2017;487:709‐715.2844234410.1016/j.bbrc.2017.04.121PMC5565483

[29] Sun T , Liu H , Ming L . Multiple roles of autophagy in the sorafenib resistance of hepatocellular carcinoma. Cell Physiol Biochem. 2017;44:716‐727.2916915010.1159/000485285

[30] Sui X , Kong N , Ye L , et al. p38 and JNK MAPK pathways control the balance of apoptosis and autophagy in response to chemotherapeutic agents. Cancer Lett. 2014;344:174‐179.2433373810.1016/j.canlet.2013.11.019

[31] Zhan Y , Gong K , Chen C , Wang H , Li W . P38 MAP kinase functions as a switch in MS‐275‐induced reactive oxygen species‐dependent autophagy and apoptosis in human colon cancer cells. Free Radic Biol Med. 2012;53:532‐543.2263414710.1016/j.freeradbiomed.2012.05.018

[32] Wang QQ , Guo XC , Li L , Gao ZH , Ji M . Treatment with metformin and sorafenib alleviates endometrial hyperplasia in polycystic ovary syndrome by promoting apoptosis via synergically regulating. Autophagy. 2019.10.1002/jcp.2905131256441

[33] Wang K . Autophagy and apoptosis in liver injury. Cell Cycle. 2015;14:1631‐1642.2592759810.1080/15384101.2015.1038685PMC4614283

